The article "Upregulated expression levels of ADAM10 and EGFR and downregulated expression levels of E-cadherin in hepatocellular carcinomas" was retracted in 2014. Reasons: errors in the data; no approval from a third party.

# Upregulated expression levels of ADAM10 and EGFR and downregulated expression levels of E-cadherin in hepatocellular carcinomas

**DOI:** 10.3892/etm.2013.1340

**Published:** 2013-10-10

**Authors:** YUAN YUE, YUMIN YANG, LEI SHI, ZUOREN WANG

**Affiliations:** 1 Department of Pharmacy, First Affiliated Hospital of Medical College of Xi’an Jiaotong University, Xi’an, Shaanxi 710061, P.R. China; 2 The Hospital of Luonan, Luonan, Shaanxi 726100, P.R. China; 3 Department of Hepatobiliary Surgery, First Affiliated Hospital of Medical College of Xi’an Jiaotong University, Xi’an, Shaanxi 710061, P.R. China

**Keywords:** hepatocellular carcinoma, ADAM10, epidermal growth factor receptor, E-cadherin

## Abstract

The aim of this study was to investigate the expression and significance of a disintegrin and metalloproteinase 10 (ADAM10), epidermal growth factor receptor (EGFR) and E-cadherin protein in hepatocellular carcinomas. The expression levels of ADAM10, EGFR and E-cadherin were analyzed in 40 cases of hepatocellular carcinoma using immunohistochemistry and quantitative polymerase chain reaction (qPCR). The expression levels of ADAM10, EGFR and E-cadherin were significantly correlated with portal vein thrombosis, intrahepatic metastasis, differentiation degree and tumor size (P<0.05). In hepatocellular carcinoma, the expression levels of ADAM10 and EGFR were increased and the levels of E-cadherin were decreased compared with those in the adjacent tissues. The elevated expression levels of ADAM10 and EGFR may be associated with the malignancy of the tumors. E-cadherin expression is negatively correlated with the degree of malignancy. The detection of ADAM10, EGFR and E-cadherin expression levels may contribute to an understanding of the oncogenesis and development of hepatocellular carcinomas.

## Introduction

The development and metastasis of primary hepatocellular carcinoma involves multiple factors, genes and processes, with an expression imbalance of numerous cellular molecules in the liver cells contributing to the malignancy process. A disintegrin and metalloproteinases (ADAMs) belong to a membrane-binding family of glycoproteins, which is involved in the processes of extracellular matrix degradation, cell adhesion and cell proliferation (1–3). ADAM10 is a member of the ADAM family and its elevated expression may be associated with the malignancy of tumors. In gastric, prostate, colon and lung cancer, as well as hematological malignancy, the expression of ADAM10 is abnormally high (4–6), although the mechanism behind this elevated expression is unclear (7). There are have been few studies concerning ADAM10 and the development mechanism of primary hepatocellular carcinoma in recent years.

The article "Upregulated expression levels of ADAM10 and EGFR and downregulated expression levels of E-cadherin in hepatocellular carcinomas" was retracted in 2014. Reasons: errors in the data; no approval from a third party.

By contrast, there have been numerous studies investigating the epidermal growth factor receptor (EGFR) and tumor development. EGFR regulates tumor cell proliferation and metastasis through the mitogen-activated protein kinase (MAPK) pathway in pancreatic and colon cancer cells (8). In prostate cancer cells, EGFR regulates cell proliferation, invasion and metastasis through the phosphoinositide 3-kinase (PI3K)/AKT pathway (9). In the development of hepatocellular carcinoma, the function of EGFR is unclear, and the proliferation of hepatocellular carcinoma may be associated with the MAPK/extracellular-signal-regulated kinase (ERK) signaling pathway (10,11).

E-cadherin is calcium-dependent cell adhesion molecule, which is believed to influence the inhibition of metastasis and is associated with the occurrence, development and clinical prognosis of a variety of types of tumor. It has been shown that in several types of tumor, including colon cancer, urinary tract tumors and oral epithelial cell carcinoma, there is a low level of or no E-cadherin expression (10,12). E-cadherin is important in the maintenance of cell integrity and polarity and the organization of structural integrity (13,14). Therefore, it has been suggested that the downregulation of E-cadherin expression promotes the invasion of tumor cells, weakening or eradicating the adhesion between these cells, and promotes the spread of the cancer cells. It has been widely observed that the level of E-cadherin expression is negatively correlated with the degree of malignancy (15).

In the present study, we collected 40 samples of primary hepatocellular carcinoma and the adjacent tissue. Using immunohistochemistry and quantitative polymerase chain reaction (qPCR), the protein and gene expression levels of ADAM10, EGFR and E-cadherin were determined, in order to investigate the correlation between their expression levels and the development of hepatocellular carcinoma.

## Materials and methods

### Patient data

Twenty samples of small hepatocellular carcinoma and the adjacent tissue were collected randomly from 30 consecutive cases of hepatocellular carcinoma. In addition, 20 samples of large hepatocellular carcinoma and the adjacent tissue were collected. Each of the 40 samples was confirmed by pathological examination (without radiotherapy and chemotherapy and prior to surgery). Of the 40 patients, there were 23 males (57.5%) and 17 females (42.5%), with an average age of 48.6 years. Following pathological identification, it was revealed that six of the cases were well differentiated (15.0%), 16 of the cases were moderately differentiated (40.0%) and 18 of the cases had a low degree of differentiation (45.0%). In addition, there were 35 cases that were positive for hepatitis B surface antigen, 29 cases of cirrhosis, and 7 cases of patients with a family history of hepatocellular carcinoma. The study was approved by the ethics review board of Xi’an Jiaotong University (Xi’an, China). Prior written and informed consent was obtained from every patient.

The article "Upregulated expression levels of ADAM10 and EGFR and downregulated expression levels of E-cadherin in hepatocellular carcinomas" was retracted in 2014. Reasons: errors in the data; no approval from a third party.

### Immunohistochemistry

ADAM10 antibody was purchased from Santa Cruz Biotechnology, Inc. (Santa Cruz, CA, USA), while EGFR and E-cadherin antibodies, streptavidin-peroxidase, 4-dimethylaminoazobenzene (DAB), the streptavidin-peroxidase immunohistochemical staining kit and normal goat serum were all purchased from Beijing Biosynthesis Biotechnology Co., Ltd. (Beijing, China). The adjacent tissue that was collected was positioned 2 cm around the cancerous tissue, and the cancerous and adjacent tissues were preserved. A positive biopsy in the kit was used for the staining of the positive control, and the antibody was replaced by phosphate-buffered saline for the staining of the negative control. Yellow to brownish-yellow granules in cells were considered to indicate positive cells. Positive cells were counted in a total of 100 cells using high-power microscopy, and scored according to the positive expression rate (0 points for <10%; 1 point for 11–20%; 3 points for 21–50%; 4 points for >50%) and staining intensity (0 points for no staining; 2 points for weak; 3 points for strong). The sum of the points for staining intensity and positive expression rate was used as the expression score. A score ≥3 was considered to indicate a positive case and a score of 0–2 was classified as a negative case.

### qPCR

Total RNA was extracted for qPCR. The primers and internal reference primers were synthesized by Shanghai Allcare Biomedical Development Co,. Ltd. (Shanghai, China) and the Ct value comparison method (16) was used to detect the gene expression level, with β-actin as an internal reference. The relative expression levels of ADAM10, EGFR and E-cadherin were calculated with the Ct value referring to the number of cycles when the fluorescence signal reached the set threshold in each reaction tube. The primers used in this study are shown in Table I.

### Statistical analysis

Data was analyzed using SPSS 16.0 statistical software (SPSS, Inc., Chicago, IL, USA). Measurement data were compared using a paired t-test, while the correlation of ADAM10, EGFR and E-cadherin expression was analyzed using Spearman’s rank correlation analysis. P<0.05 was considered to indicate a statistically significant difference.

## Results

### Protein expression of ADAM10, EGFR and E-cadherin

To detect the expression ADAM10, EGFR and E-cadherin proteins, immunohistochemical analyses of ADAM10, EGFR and E-cadherin expression in hepatocellular carcinomas and their adjacent tissues were performed (Fig. 1). It was shown that ADAM10 and EGFR were expressed in hepatocellular carcinoma and the adjacent tissues. The positive expression rates and scores of ADAM10 and EGFR were significantly increased in the cancerous tissue compared with those in the adjacent tissue (P<0.05). E-cadherin was also expressed in hepatocellular carcinoma and the adjacent tissues; however, the positive expression rates and scores of E-cadherin were significantly increased in the adjacent tissues compared with those in hepatocellular carcinoma (P<0.05; Table II and Fig. 1). These results indicate that in hepatocellular carcinoma, the expression levels of ADAM10 and EGFR are increased and the levels of E-cadherin are decreased compared with those in adjacent tissues.

The article "Upregulated expression levels of ADAM10 and EGFR and downregulated expression levels of E-cadherin in hepatocellular carcinomas" was retracted in 2014. Reasons: errors in the data; no approval from a third party.

### mRNA levels of ADAM10, EGFR and E-cadherin

To detect the possible changes in the mRNA levels of ADAM10, EGFR and E-cadherin expression in hepatocellular carcinoma and the adjacent tissues, qPCR was performed. The qPCR results showed significant gene expression level differences between the cancerous and adjacent tissues (P<0.05). The expression of ADAM10 and EGFR in the cancerous tissue was significantly increased (P<0.05) while the E-cadherin mRNA expression in the cancerous tissue was significantly decreased compared with that in the adjacent tissue (P<0.05), as shown in Table III and Fig. 2. These results indicate that in hepatocellular carcinoma, the mRNA levels of ADAM10 and EGFR are increased and the mRNA levels of E-cadherin are decreased compared with those in the adjacent tissues.

### Correlation between the protein and gene expression of ADAM10, EGFR and E-cadherin and the clinical pathology examination results

To investigate the correlation between the protein expression and mRNA levels of ADAM10, EGFR and E-cadherin and the clinical pathology examination results, the positive protein expression scores were analyzed (Table IV). It was revealed that ADAM10 and EGFR were positively correlated with a correlation coefficient of 0.7152, while ADAM10 and E-cadherin were negatively correlated, with a correlation coefficient of −0.6149. In the 40 cases of liver cancer, the protein expression of ADAM10, EGFR and E-cadherin protein in the cancer tissue was not significantly correlated with gender or age. However, there were significant differences in the protein expression levels between: tissues with a low degree of differentiation and those with a moderate/high degree of differentiation; tumors with diameters of < and >5 cm; tumors with and without portal vein thrombosis; and tumors with and without intrahepatic metastasis (P<0.05). Similar results were obtained for the gene expression levels. The mRNA expression levels of ADAM10 and EGFR were positively correlated, with a correlation coefficient of 0.6848, while the mRNA expression levels of ADAM and E-cadherin were negatively correlated, with an expression correlation coefficient of −0.6052. In the 40 samples of hepatocellular carcinoma, there was no significant correlation between mRNA expression and patient gender or age. However, there were significant differences in mRNA expression levels between: tissues with a low degree of differentiation and those with a moderate/high degree of differentiation; tumors with diameters of < and >5 cm; tumors with and without portal vein thrombosis; and tumors with and without intrahepatic metastasis (P<0.05). These results suggest that the elevated expression of ADAM10 and EGFR may be correlated with the malignancy of tumors and that E-cadherin expression may be negatively correlated with the degree of malignancy.

The article "Upregulated expression levels of ADAM10 and EGFR and downregulated expression levels of E-cadherin in hepatocellular carcinomas" was retracted in 2014. Reasons: errors in the data; no approval from a third party.

## Discussion

In this study, the ADAM10 protein expression level was detected in cancer and adjacent tissue using immunohistochemistry. The immunohistochemical analysis showed that the ADAM10 protein level was increased in the cancer tissue compared with that in the adjacent tissue (P<0.05), which indicated the correlation between a high expression level of ADAM10 and cancer formation. In a previous study, Liu *et al*(17) described the elevated expression of ADAM10 in breast cancer tissue and applied ADAM10 inhibitors to inhibit epidermal growth factor release and tumor cell proliferation. Consistent with this, Gavert *et al*(4) revealed that there was an elevated expression of ADAM10 in colon cancer tissue and suggested that increased levels of ADAM10 promoted colon cancer liver metastases. In the present study, qPCR was used to show that the mRNA expression of ADAM10 was increased in the cancer group compared with that in the adjacent group (P<0.05). The elevated mRNA and protein levels were consistent with each other. In a study by Rocks *et al*(18), it was demonstrated that ADAM10 gene expression level was significantly increased in non-small cell lung cancer compared with that in normal tissue. In the 40 hepatocellular carcinoma samples of the current study, the ADAM10 mRNA and protein expression levels were significantly increased in the tissue from large (>5 cm) hepatocellular carcinoma compared with those in the tissue from small hepatocellular carcinomas. Furthermore, the mRNA and protein expression levels were increased in tissue with intrahepatic metastasis compared with those without intrahepatic metastasis. This suggests that ADAM10 was important in the promotion of the proliferation and metastasis of hepatocellular carcinoma. The ADAM10 protein expression levels in hepatocellular carcinoma were significantly correlated with the gene transcription levels.

The article "Upregulated expression levels of ADAM10 and EGFR and downregulated expression levels of E-cadherin in hepatocellular carcinomas" was retracted in 2014. Reasons: errors in the data; no approval from a third party.

In this study, following the detection of E-cadherin gene and protein expression levels, it was observed that the expression level of E-cadherin was significantly reduced in cancer tissue (P<0.05). The expression level was correlated with degree of differentiation, with the expression being lower in the group with the low degree of differentiation compared with that in the highly differentiated group (P<0.05). This suggests that the E-cadherin expression level decreased with the degree of malignancy. The decreased expression of E-cadherin may be an important biological indicator of the degree of malignancy in hepatocellular carcinoma and may be used for the determination of recurrence and metastasis (19).

In this study, it was shown that the E-cadherin protein expression level was decreased in cancer tissue, while EGFR protein expression level was increased in cancer tissue. This suggested the occurrence of a mutual regulation of E-cadherin and EGFR on the cell surface. The ADAM10 expression level in hepatocellular carcinoma was positively correlated with EGFR protein expression and negatively correlated with E-cadherin protein expression, indicating that ADAM10 was involved in the regulation of EGFR and E-cadherin expression. In the planned follow-up experiment, ADAM10 gene expression level was downregulated, in order to observe the gene and protein expression levels of EGFR and E-cadherin and the influence of the downregulated ADAM10 gene expression level on the proliferation, invasion and migration of the cancer cell line HepG2. In conclusion, the elevated expression of ADAM10 and EGFR may be associated with the malignancy of tumors. E-cadherin expression was negatively correlated with the degree of malignancy. The detection of ADAM10, EGFR and E-cadherin may contribute to an understanding of the oncogenesis and development of hepatocellular carcinomas.

## Figures and Tables

**Figure 1:** Immunohistochemical analysis of a disintegrin and metalloproteinase 10 (ADAM10), epidermal growth factor receptor (EGFR) and E-cadherin expression in hepatocellular carcinoma and the adjacent tissue (magnification, ×200). A positive biopsy in the kit was used for the staining of the positive control and the antibody was replaced by phosphate-buffered saline for the staining of the negative control. Yellow to brownish-yellow granules in the cells were considered to indicate positive cells. Positive cells were counted in a total of 100 cells using high-power microscopy, and scored according to the positive expression rate (0 points for <10%; 1 point for 11–20%; 3 points for 21–50%; 4 points for >50%) and staining intensity (0 points for no staining; 2 points for weak; 3 points for strong). The sum of the points for staining intensity and positive expression rate was used as the expression score. A score ≥3 was considered to indicate a positive case and a score of 0–2 was classified as a negative case.

The article "Upregulated expression levels of ADAM10 and EGFR and downregulated expression levels of E-cadherin in hepatocellular carcinomas" was retracted in 2014. Reasons: errors in the data; no approval from a third party.

**Figure 2:** Quantitative polymerase chain reaction (qPCR) results. Total RNA was extracted. The primers and internal reference primers were synthesized by the Shanghai Allcare Biomedical Development Co,. Ltd. (Shanghai, China) and the Ct value comparison method was used to detect the gene expression level with β-actin as internal reference. The relative expression levels of a disintegrin and metalloproteinase 10 (ADAM10), epidermal growth factor receptor (EGFR) and E-cadherin were calculated with the Ct value referring to the number of cycles when the fluorescence signal reached the set threshold in each reaction.

**Table I:** Primers used in this study.

Primers	Sequences
ADAM10	F: 5′-TGGCTCATTGGTGGGCAGTATTAC-3′
	R: 5′-TGGTTTAGGAGGCAACTTTGG-3′
EGFR	F: 5′-GGTGGCTGGTTATGTCCTCATTG-3′
	R: 5′-AGTTTCTGGCAGTTCTCCTCTC-3′
E-cadherin	F: 5′-AGCGTGTGTGACTGTGAAGG-3′
	R: 5′-GCTGGCTCAAGTCAAAGTCC-3′
β-actin	F: 5′-CGACAGGATGCAGAAGGAGA-3′
	R: 5′-CGTCATACTCCTGCTTGCTG-3′

ADAM, a disintegrin and metalloproteinase; EGFR, epidermal growth factor receptor; F, forward; R, reverse.

**Table II:** ADAM10, EGFR and E-cadherin expression in hepatocellular carcinoma and adjacent tissue.

		ADAM10		EGFR		E-cadherin	
				
Tissue type	n	Positive cases n (%)	Expression score (mean ± SD)	Positive cases n (%)	Expression score (mean ± SD)	Positive cases n (%)	Expression score (mean ± SD)
Cancer tissue	40	33 (82.5)	4.19±1.88	37 (92.5)	3.21±2.01	12 (30.0)	2.08±1.40
Adjacent tissue	40	7 (17.5)	2.58±0.54	14 (35.0)	2.24±0.96	24 (60.0)	3.24±1.72

Differences in the expression levels of three proteins between the cancer and adjacent tissues are significant (P<0.05). ADAM, a disintegrin and metalloproteinase; EGFR, epidermal growth factor receptor; SD, standard deviation.

**Table III:** mRNA expression of ADAM10, EGFR and E-cadherin in hepatocellular carcinoma and adjacent tissue.

Tissue type	n	ADAM10	EGFR	E-cadherin
Cancer tissue	40	0.753±0.214	0.623±0.178	0.213±0.058
Adjacent tissue	40	0.346±0.231	0.378±0.092	0.552±0.151

Values presented are the mean ± standard deviation. Differences in the expression levels of three genes between the cancer and adjacent tissues are significant (P<0.05). ADAM, a disintegrin and metalloproteinase; EGFR, epidermal growth factor receptor.

The article "Upregulated expression levels of ADAM10 and EGFR and downregulated expression levels of E-cadherin in hepatocellular carcinomas" was retracted in 2014. Reasons: errors in the data; no approval from a third party.

**Table IV:** Correlation between the protein/mRNA expression of ADAM10, EGFR and E-cadherin and clinical pathology in 40 cases of liver cancer.

		ADAM10		EGFR		E-cadherin	
				
Factors	Cases	Protein expression score	mRNA relative value	Protein expression score	mRNA relative value	Protein expression score	mRNA relative value
Gender							
Male	23	4.11±1.42	0.762±0.252	3.35±2.28	0.668±0.169	2.17±1.21	0.227±0.105
Female	17	4.44±1.35	0.711±0.205	3.15±2.21	0.619±0.154	2.02±1.01	0.203±0.112
Age (years)							
>50	24	4.27±1.49	0.741±0.213	3.11±2.75	0.631±0.177	2.04±1.98	0.235±0.207
≤50	16	4.05±1.32	0.771±0.221	3.41±2.04	0.622±0.152	2.11±1.06	0.195±0.174
Tumor size (cm)							
>5	20	4.85±0.65^a^	0.784±0.252^a^	4.19±2.24^a^	0.793±0.255^a^	0.64±0.25^a^	0.187±0.167^a^
<5	20	2.89±1.58	0.612±0.198	2.25±1.98	0.594±0.162	2.64±1.69	0.305±0.250
Portal vein thrombosis							
With	10	4.78±1.89^a^	0.812±0.311^a^	4.78±3.56^a^	0.786±0.311^a^	0.84±0.55^a^	0.174±0.132^a^
Without	30	2.72±1.38	0.665±0.173	2.79±2.73	0.582±0.194	2.98±0.51	0.312±0.241
Differentiation degree							
High and moderate	22	2.39±1.51^a^	0.610±0.114^a^	2.22±2.43^a^	0.527±0.199^a^	2.77±1.36^a^	0.298±0.178^a^
Low	18	4.72±0.92	0.871±0.294	4.01±3.72	0.775±2.123	0.85±1.02	0.201±0.105
Intrahepatic metastasis							
With	12	4.86±1.78^a^	0.901±0.225^a^	3.94±3.01^a^	0.811±0.342^a^	0.78±0.12^a^	0.112±0.054^a^
Without	28	2.76±1.73	0.678±0.223	2.55±2.43	0.551±0.162	2.75±1.13	0.376±0.223
HBV related liver cancer							
With	30	4.14±1.25	0.744±0.235	3.33±2.45	0.624±0.215	2.04±1.32	0.219±0.191
Without	10	4.37±1.03	0.775±0.247	3.07±2.75	0.632±0.244	2.12±1.01	0.204±0.147

Values presented are the mean ± standard deviation. ADAM, a disintegrin and metalloproteinase; EGFR, epidermal growth factor receptor; HBV, hepatitis B virus.

a P<0.05.
